This article has been retracted.

# MiR‐191‐5p inhibits lung adenocarcinoma by repressing SATB1 to inhibit Wnt pathway

**DOI:** 10.1002/mgg3.1043

**Published:** 2019-11-13

**Authors:** Lai‐yong Zhou, Fu‐wei Zhang, Jian Tong, Fang Liu

**Affiliations:** ^1^ Department of Cardiothoracic surgery The People's Hospital of Bao’an Shenzhen The Affiliated Bao’an Hospital of Southern Medical University Shenzhen China; ^2^ Department of Cardiothoracic surgery Zhujiang Hospital Southern Medical University Guangzhou China; ^3^ Department of Pathology The People's Hospital of Bao’an Shenzhen The Affiliated Bao’an Hospital of Southern Medical University Shenzhen China

**Keywords:** lung adenocarcinoma, metastatic lung cancer, miR‐191‐5p, *SATB1*

## Abstract

**Background:**

To investigate the function of miR‐191‐5p in lung adenocarcinoma and its possible mechanism.

**Methods:**

QRT‐PCR was adopted for the detection of the expression levels of miR‐191‐5p and *SATB1* (HGNC: 10541). The effects of miR‐191‐5p and *SATB1* on cell proliferation and migration were examined through the CCK‐8 and Transwell assays. Subsequently, the binding relationships between miR‐191‐5p and *SATB1* were confirmed by dual‐luciferase reporter gene assay. Finally, the potential mechanisms of action of miR‐191‐5p were explored through a serious of in vivo and in vitro experiments.

**Results:**

Lung adenocarcinoma patients had a notably lower expression level of miR‐191‐5p than controls, patients with metastasis had a lower level than those without metastasis, and the level in patients with lung adenocarcinoma in stage III‐IV was lower than that in patients with lung adenocarcinoma in stage I‐II. Overexpression of miR‐191‐5p repressed the migration and proliferation of lung cancer A549/H1650 cells. According to the reporter gene assay, miR‐191‐5p could bind to *SATB1*. Besides, *SATB1* was significantly overexpressed in cancer tissues of patients with lung adenocarcinoma, and *SATB1* overexpression accelerated the migration and proliferation of A549/H1650 cells and reversed inhibition on cell migration and proliferation by miR‐191‐5p.

**Conclusion:**

Overexpression of miR‐191‐5p is capable of blocking the migration and proliferation of lung cancer cells, and its mechanism may be through targeting *SATB1* thus downregulating Wnt signaling.

## Graphical abstract

MiR‐191‐5p has a notably low expression in Lung adenocarcinoma patients. MiR‐191‐5p inhibits the migration and proliferation of lung cancer cells. MiR‐191‐5p reduces the expression of SATB1 and inhibits the activation of Wnt/β‐catenin signaling pathway through its target gene SATB1.

## 1 INTRODUCTION

Lung cancer is the leading cause of cancer‐related deaths worldwide, and there are approximately 1.4 million new cases of lung cancer every year (Jemal et al., 2011) (Wei, Tian, Song, Wu, & Liu, 2018). Two major lung cancer subtypes are small cell lung cancer (SCLC) and non–small cell lung cancer (NSCLC), with the proportion of about 15%–20% and 80%–85%, respectively (Goldstraw et al., 2011). Adenocarcinoma takes up over 50% in NSCLC. In spite of therapies for lung adenocarcinoma, lung adenocarcinoma‐induced mortality rate is still high (Diaz‐Garcia et al., 2013; Rosell, Bivona, & Karachaliou, 2013), which may be associated with early metastasis (Peters et al., 2012). Hence, seeking novel targets and prognostic biomarkers is of profound significance.

microRNAs (miRNAs) are small noncoding RNA molecules modulating posttranscriptional protein expression through complementary base pairing (Lau, Lim, Weinstein, & Bartel, 2001). miRNAs are involved in tumor formation, invasion, migration, and metastasis through a variety of signaling pathways, revealing roles as therapeutic targets in cancer (Pfeffer, Yang, & Pfeffer, 2015; Rupaimoole & Slack, 2017). As the gene sequencing technology advances, miRNA expressions in lung cancer tissues and paracancerous tissues have been examined (Puissegur et al., 2011). miR‐191‐5p is known to be dysregulated in several tumors, including intrahepatic cholangiocarcinoma, breast cancer, and colorectal cancer (Li et al., 2017; Mar‐Aguilar et al., 2013; Zhang et al., 2015). However, miR‐191‐5p's function in lung adenocarcinoma remains largely unknown.

The aim of this study was to investigate the expression level of miR‐191‐5p and its potential as a therapeutic target in lung cancer. We performed analysis in patient primary adenocarcinoma tissues, cell lines, and a mouse xenograft model. Our study revealed miR‐191‐5p's therapeutic effects on inhibiting cancer cell migration and proliferation and further identified its target gene *SATB1* (HGNC: 10541) and downstream pathway.

## 2 METHODS

### 2.1 Ethical compliance

The research was approved by the Ethics Committee of The People's Hospital of Bao'an Shenzhen.

### 2.2 General data

Fresh lung adenocarcinoma and lung adenocarcinoma‐adjacent tissue samples of 24 lung adenocarcinoma patients receiving surgical treatment were collected, and the lung adenocarcinoma‐adjacent tissues should be at more than 5 cm from the edge of the tumor tissues. Besides, these patients had no history of other primary secondary tumors and no history of chemotherapy, radiotherapy, targeted therapy, etc. After collection, the samples were placed in a freezing storage tube, marked with sample information and stored in liquid nitrogen, and procedures in the whole storage and transportation process were operated under the condition with no enzyme. Meanwhile, clinicopathological data, including gender, age, smoking history, the tumor size, histological grades, pathological subtypes, TNM stages, and the lymph node status, of all the patients were collected. All the patients voluntarily entered into this research and signed the written informed consent, and this research gained the approval of the Ethics Committee of the People's Hospital of Bao'an Shenzhen.

### 2.3 Cell culture

HBE, a normal bronchial epithelial cell line, and SPC‐A1, H460, H1650, and A549, NSCLC cell lines, were all bought from ATCC. These cells were cultured in DMEM (Thermo Fisher Scientific) with RPMI‐1640 medium (Gibco‐BRL; Thermo Fisher Scientific) or 10% fetal bovine serum (FBS; Hyclone) in a constant temperature incubator with saturated humidity and 5% CO_2_ at 37°C.

### 2.4 Cell transfection

At 1 day before transfection, an appropriate number of cells were inoculated into 6‐well plates and cultured in the cell culture medium without antibiotics, followed by transient transfection when the cells filled 60%–70% of the culture dish overnight. Then the cells were transfected with miR‐191‐5p mimics, pcDNA‐SATB homeobox 1 (*SATB1*) and corresponding negative controls and mixed with Lipo2000. Subsequently, the mixture was let stand for 20 min after even mixing at room temperature to form the DNA/Lipo2000 (or mimics/Lipo2000) complex. 100 μL of the complex was slowly dripped into the culture solution and mixed well to co‐culture the cells for 4–6 hr. Thereafter, the complex was discarded, and the complete culture medium containing 1% streptomycin and 10% FBS was used to replace the culture medium for 24 hr for subsequent experiments.

### 2.5 Extraction of total RNA from tissues and cells

About 50 mg tissues were taken, ground in liquid nitrogen, and added with 1 ml TRIzol (Invitrogen). Then cells were washed with PBS once after collection, added with 1 ml TRIzol at the cell density of 5 × 10^6^/ml. After that, the tissues or cells were fully homogenized, transferred to a 1.5 ml centrifuge tube, and let stand for 5 min. Chloroform with a volume 0.2 times that of the volume of TRIzol (TRIzol: chloroform = 1:0.2) was added into a centrifuge tube containing lysate and let stand for 5 min at room temperature after even mixing, followed by 10 min of centrifugation. Then the supernatant was transferred to another unused 1.5 ml centrifuge tube, and the DNaseI (RNase Free, TaKaRa) was applied to remove the residual DNAs according to manual. Afterward, the supernatant was added with an equal volume of isopropyl alcohol, mixed evenly and centrifuged for 10 min, and ultimately the supernatant was carefully sucked and discarded. After that, a centrifuge tube containing RNA precipitates was added with 1 ml of 75% ethanol, mixed uniformly, let stand at room temperature for 5 min, and centrifuged for 5 min. Finally, the supernatant was carefully sucked and discarded, and the RNA precipitates were dried at room temperature and dissolved in diethyl pyrocarbonate (DEPC)‐treated water based on their amount.

### 2.6 Quantitative reverse transcription‐polymerase chain reaction (qRT‐PCR)

After the test of purity and concentration of RNA samples, cDNA samples were synthesized by RT, with GAPDH and U6 as the internal references. DEPC (Beyotime Biotechnology), SYBR Green (Applied Biosystems) premixed solution, forward (F)/reverse (R) primers, and templates were prepared into PCR solution, which was placed on a RT‐PCR instrument for PCR amplification. miRNAs were reversely transcribed into cDNAs by miRNA RT kit [Tiangen Biotech (Shanghai) Co., Ltd.], and PCR and quantitative analysis of miRNAs were carried out according to miRNA qPCR kit instructions [Tiangen Biotech (Shanghai) Co., Ltd.]. Primer sequences are listed below:

miR‐191‐5p (F: 5′ CAACGGAATCCCAAAAGCAGCTG 3′,

R: As provided by the miScript SYBR Green kit;

U6 (F: 5′ CTCGCTTCGGCAGCACA 3′, R: 5′ ACGCTTCACGAATTTGCGT 3′);

GAPDH (F: 5' GAAGGTGAAGGTCGGAGTC′, R: 5′ GAAGATGGTGATGGGATT TC′);

*SATB1* (F: 5′ GATCATTTGAACGAGGCAACTCA 3′, R: 5′ TGGACCCTTCGGATC

ACTCA 3′)

#### 2.6.1 Luciferase enzyme detection

The sequence of the 3'UTR of *SATB1* transcripts was cloned into the vector pGL3 containing luciferase reporter genes as WT3'UTR group. The key binding region of miRNAs on the 3'UTR mutated into invalid binding sequences using the site‐directed mutagenesis kit to form control plasmid MUT3′UTR group. Each group was transfected with miR‐191‐5p mimics and marine kidney luciferase plasmids (internal reference). After transfection for 24 hr, the cell culture solution was aspirated completely. According to the requirements of the kit, an appropriate amount of lysate was added to fully lyse the cells. Following centrifugation, 100 μL of the supernatant of the lysate was harvested for determination. The RLU value determined by firefly luciferase was divided by that determined by *renilla* luciferase with *renilla* luciferase as internal reference. According to the obtained ratio, the activation degree of different sample target reporter genes was compared.

### 2.7 Cell migration

A Transwell chamber was placed above a 24‐well plate. After trypsinization, the transfected NSCLC cells were suspended in serum‐free medium, followed by counting with a cell counting plate. After that, the cells were diluted with serum‐free medium, whose density was adjusted to 1 × 10^5^/ml, and the chamber was added with the above cell suspension. Then the cells in the sterile 24‐well plate was added with a culture medium with 10% FBS in an incubator for incubation. 48 hr later, the culture medium was discarded, followed by washing with PBS, and the Transwell chamber was taken out and fixed with 4% paraformaldehyde for 30 min. After staining with 0.5% crystal violet added for 10–15 min, the staining agent was rinsed with PBS. Finally, observation and counting of the cells were performed using a microscope.

### 2.8 Cell proliferation

NSCLC cells after treatment were inoculated into 96‐well plates (1 × 10^4^/well), followed by culture for 0 hr, 24 hr, 48 hr, and 72 hr, respectively. Cell Counting Kit‐8 (CCK‐8) kit (Dojindo) was utilized to detect the cell proliferation ability, before which CCK‐8 and the culture medium were mixed at 1:10 to prepare a mixed solution. The culture medium used previously was discarded, and 110 μL of the mixed culture medium was added for further 1 hr of incubation at 37°C away from light. Ultimately, the OD value at 450 nm was examined by ELISA, and six replicate wells were set in each group.

### 2.9 Western blotting

Through centrifugation at 12,000 × g and 4°C for 20 min, total proteins were extracted, whose concentration was evaluated by BCA protein assay kit (Beyotime). After that, the same quantities of total proteins were isolated in 10% SDS‐PAGE and transferred onto nitrocellulose membranes, which were then sealed with 5% skim milk powder in TBS containing 0.5% Tween‐20 for 1 hr. Afterward, a primary antibody was added for incubation at 4°C overnight, and the proteins were rinsed and incubated with a secondary antibody for 2 hr at room temperature. Eventually, ECL and Western blotting detection reagents (Thermo Fisher Scientific, Inc.) were employed to examine the membranes. The above antibodies (Abcam) were utilized by reference to the manufacturer's instructions.

### 2.10 Tumor growth assay in vivo

Animal experiments gained the approval of the Animal Use and Care Committee of Jiangsu University. A total of six male BALB/c nude mice aged 4 weeks old were allocated into two groups randomly. At 36 hr after transfection, A549 cells subjected to transfection with miR‐191‐5p agomir and NC were obtained, and 0.2 ml PBS was utilized to resuspend about 2 × 10^6^ A549 cells, which were then injected into each mouse subcutaneously. After cell inoculation, xenografts were periodically observed. At 6 weeks after injection, these mice were executed, followed by the removal and photographing of xenografts. Ultimately, a vernier caliper was applied to measure the tumor diameter, and the tumor volume (V) was calculated based on the formula:

### 2.11 Immunohistochemical staining

Anti‐Ki‐67 primary monoclonal antibody (Cell Signaling Technology) was added to incubate tumor tissue sections, which were subjected to further incubation with the secondary antibody at room temperature for 30 min. Following 5 min of incubation with 3,3'‐DAB (Maxim), 30 s of counterstain of the sections was carried out with hematoxylin, followed by photographing under a TE2000 microscope (Nikon).

### 2.12 Statistical methods

SPSS 23.0 (SPSS, Inc.) was adopted for data statistical processing. χ^2^ test was carried out to compare count data, and comparisons of measurement data were detected via the independent samples *t*‐test between the two groups. *p* < .05 represented that the difference was of statistical significance.

## 3 RESULTS

### 3.1 miR‐191‐5p exhibited an significantly low expression in lung cancer cell lines

At first, miR‐191‐5p expression levels in lung cancer tissues and corresponding cancer‐adjacent tissues were measured, the results of which revealed that miR‐191‐5p was significantly lowly expressed in lung cancer tissues (Figure 1a). Second, the expression of miR‐191‐5p in different lung cancer stages were detected, which manifested that miR‐191‐5p expression in patients with lung cancer in stage III‐IV was markedly lower than that in patients with cancer in stage I‐II (Figure 1b). Thirdly, lung cancer group was subdivided into metastasis group and nonmetastasis group, and miR‐191‐5p expression levels in the two groups were examined. According to the results, miR‐191‐5p exhibited a notably low expression in the tissues of patients with cancer metastasis (Figure 1c). Ultimately, the survival analysis displayed that patients with lowly expressed miR‐191‐5p had significantly lower survival rates than those with highly expressed miR‐191‐5p (Figure 1d). The above results indicate that miR‐191‐5p may exert certain effects in the process of lung cancer.

**Figure 1:** miR‐191‐5p expression level correlates with lung cancer metastasis in patient tissue samples. (a) miR‐191‐5p expression significantly declined in lung cancer tissues compared with that in paracancerous tissues. (b) miR‐191‐5p expression in the tissues of patients with lung cancer in stage III‐IV is remarkably lower than that in patients with lung cancer in stage I‐II. (c) miR‐191‐5p expression in metastasis group is lower than that in non‐metastasis group. (d) Survival analysis reveals that patients with low miR‐191‐5p expression have lower survival rates than those with high expression. ***p < .001

### 3.2 miR‐191‐5p could inhibit cell proliferation and migration

In addition, miR‐191‐5p expression level in lung cancer cell lines was also determined. According to the results, compared with that in HBE, miR‐191‐5p expression level was generally lower in lung cancer cell lines (Figure 2a). To elaborate the possible role of miR‐191‐5p in lung cancer's occurrence and development, A549 and H1650 cells were chosen for the following research. After transfection with miR‐191‐5p mimics, miR‐191‐5p expressions in the two cell lines were elevated in comparison with that in control group (Figure 2b). The functions of miR‐191‐5p expression in cell proliferation and migration were examined through the upregulation of its expression. The results denote that cell migration and proliferation are markedly repressed after an increase in miR‐191‐5p expression (Figure 2c‐f).

**Figure 2:** miR −191‐5p inhibits cell proliferation and migration. (a) In comparison with that in normal bronchial epithelial cells, miR‐191‐5p expression is generally downregulated in lung cancer cell lines. (b) After A549 and H1650 cells are transfected with miR‐191‐5p mimics, miR‐191‐5p expression is markedly elevated. (c,d) Cell proliferation ability is significantly inhibited after miR‐191‐5p expressions in A549 and H1650 cells are elevated. (e,f) Cell migration ability is remarkably inhibited after miR‐191‐5p expressions in A549 and H1650 cells are increased. *p < .05, **p < .01, ***p < .001

### 3.3 *SATB1* was a potential target gene of miR‐191‐5p

Prediction and analysis through websites illustrated that *SATB1* was a potential target gene of miR‐191‐5p (Figure 3a), and the dual‐luciferase reporter gene assay further confirmed the binding relationship between the two (Figure 3b,c). *SATB1* expression was measured after overexpression of miR‐191‐5p in A549 and H1650 cells, which displayed that both mRNA and protein expression levels of *SATB1* were remarkably inhibited (Figure 3d‐f). The above results denote that *SATB1* is the target gene of miR‐191‐5p, and miR‐191‐5p can reduce *SATB1* expression.

**Figure 3:** *SATB1* is a potential target gene of miR‐191‐5p. (a) Bioinformatics analysis shows that the two have potential binding sites. (b,c) Dual‐luciferase reporter gene displays that there is a binding relationship between them. (d‐f) Following miR‐191‐5p expressions in A549/H1650 cells are increased, *SATB1* expression is notably decreased. **p < .01, ***p < .001

### 3.4 *SATB1* could promote cell proliferation and migration

Since *SATB1* is a target gene of miR‐191‐5p, its expression in tissues of lung cancer patients was examined. It was discovered that cancer tissues had prominently higher *SATB1* expression than adjacent tissues (Figure 4a). According to Pearson correlation analysis, miR‐191‐5p had a negative relationship to *SATB1* expression in lung cancer tissues (*r^2^* = 0.352, *p* = .0022) (Figure 4b). After A549 and H1650 cells were transfected with *SATB1* overexpression plasmids, *SATB1* expression was notably elevated (Figure 4c). The results of CCK‐8 and Transwell assays illustrated that the upregulation of *SATB1* expression remarkably accelerated the migration and proliferation of lung cancer cells (Figure 4d‐f).

**Figure 4:** *SATB1* can promote cell proliferation and migration. (a) Compared with that in cancer‐adjacent tissues, *SATB1* is significantly highly expressed in lung cancer tissues. (b) Pearson analysis validates that a negative correlation exists between the two expressions. (c) After A549 and H1650 cells are transfected with *SATB1* plasmids, *SATB1* expressions are markedly elevated. (d‐f) The elevated *SATB1* expressions in A549/H460 cells can promote the cell proliferation and migration ability. *p < .05, **p < .01, ***p < .001

### 3.5 miR‐191‐5p exerted its effects by decreasing ***SATB1***

After *SATB1* overexpression in A549 and H1650 cells, β‐catenin expression level was significantly raised (Figure 5a). Increased miR‐191‐5p suppressed β‐catenin expression, but elevated *SATB1* partially restored it (Figure 5b). Furthermore, in order to explore whether miR‐191‐5p exerts its effects by decreasing *SATB1*, a rescue experiment was carried out. The experimental results confirmed that the migration and proliferation abilities of A549 and H1650 cells were prominently weakened after an increase in miR‐191‐5p expression. However, the proliferation and migration abilities of cells were partially improved after the expressions of both miR‐191‐5p and *SATB1* were elevated (Figure 5c‐e), which indicates that miR‐191‐5p reduces the expression of *SATB1* and inhibits the activation of Wnt/β‐catenin signaling pathway through its target gene *SATB1*.

**Figure 5:** miR −191‐5p exerts its effects by decreasing *SATB1.* (a) The expression of β‐catenin is notably increased after upregulation of *SATB1* in cells. (b) The expression of β‐catenin is markedly reduced after overexpression of miR‐191‐5p in cells, which partially restores the expression of β‐catenin. (c‐e) Upregulation of *SATB1* partially reverses the inhibitory effect of miR‐191‐5p on cell migration and proliferation. *p < .05, **p < .01

### 3.6 miR‐191‐5p inhibited tumor growth

The roles of miR‐91‐5p in lung cancer in vivo were discussed by construction of a mouse model of xenograft. Six weeks later, the mice treated with miR‐191‐5p agomir cells formed significantly smaller tumors than those treated with NC, as determined by tumor size and weight (Figure 6a‐c). It was also discovered that miR‐191‐5p was over‐expressed in the miR‐191‐5p agomir‐injected tumor sections than NC‐injected tumor sections (Figure 6d). Furthermore, to indicate the proliferation of intratumoral cells, immunohistochemical method was used for detecting the expression of intratumoral Ki67, a marker of cell proliferation, in each group. The results indicated that Ki67 positive staining showed brown‐yellow granules, and the number of Ki67‐positive expression cells and their degree of positive staining in tumor tissues were reduced in miR‐191‐5p‐A549‐injected mice, indicating that miR‐191‐5p treatment slows the proliferation of intratumoral cells to some extent (Figure 6e,f).

**Figure 6:** miR‐191‐5p inhibits tumor growth. (a‐c) Tumor volumes and weights of mice in mir‐191‐5p and NC groups. (d) QRT‐PCR analysis of miR‐191‐5p expression in tissues of resected tumors. (e,f) Typical images of HE staining and immunohistochemical staining of Ki‐67 in mouse tumor tissues. Original magnification: ×100. **p < .01, ***p < .001

## 4 DISCUSSION

The implication of miRNAs in tumorigenesis was first recognized when miRNA genes were observed to be specifically deleted in patients with leukemia (Dyrskjot et al., 2009). There is increasing evidence that miRNAs are related to tumor aggressiveness and metastatic potential and are considered diagnostic and prognostic markers for multiple cancers, including lung cancer (Dai et al., 2019; Dong, Li, & Wang, 2019).

The function of miR‐191‐5p differs among different tumors. According to one study on ovarian cancer, miR‐191‐5p inhibits apoptosis induced by TNF‐α in endometrial carcinoma cells by targeting DAPK1 (Tian, Xu, & Wang, 2015). Additionally, miR‐191‐5p could promote the tumorigenesis of colorectal cancer by targeting CCAAT‐enhancer‐binding protein β (Zhang et al., 2015). In lung cancer, inhibition of miR‐191 contributes to radiation‐resistance of two lung cancer cell lines by altering autophagy activity (Liu & Huang, 2015). However, another study revealed that overexpression of miR‐191 does not lead to an alteration in cell cycle, proliferation, and chemosensitivity of A549 and BEAS‐2B cell lines (Patnaik, Kannisto, & Yendamuri, 2010). Meanwhile, it was also found that the expression of miR‐191 was significantly upregulated in NSCLC cells in patients in vivo (Zhang, Ma, Zhang, Huo, & Zhao, 2017). Therefore, the effects of miR‑191 in the development of lung cancer are still a subject of debate. It was discovered in this research that miR‐191‐5p was lowly expressed in lung adenocarcinoma and lung cancer cell lines. It has not ever been reported before. The results of experiments in vitro and in vivo revealed that miR‐191‐5p could repress the migration and proliferation of A549/H1650 cells, furtherly, blocked the growth of tumor. Therefore, miR‐191‐5p may act as a tumor suppressor in lung adenocarcinoma cancer.

In order to further unfold the potential mechanism of action of miR‐191‐5p, the bioinformatics analysis was performed, which revealed that *SATB1* was its potential target gene, which was validated by dual‐luciferase reporter gene assay. *SATB1*, a nuclear matrix‐associated protein, adjusts the expression of multiple genes by functioning in chromatin remodeling mechanisms (Kohwi‐Shigematsu et al., 2013; Nodin et al., 2012). *SATB1* interacts with the Wnt‐β‐catenin pathway (Gattinoni, Ji, & Restifo, 2010) and is also correlated with many types of cancers (Elebro et al., 2014; Selinger et al., 2011). It is known that Wnt/β‐catenin signaling adjusts numerous cellular processes, including proliferation, invasion and differentiation, by adjusting the ability of the multifunctional β‐catenin protein, which is a vital signaling molecule in the Wnt/β‐catenin pathway (Javed et al., 2019; Zhan, Rindtorff, & Boutros, 2017).

In this research, the expression of *SATB1* in lung cancer was assessed, which demonstrated that *SATB1* exhibited a high expression in lung cancer tissues and was negatively related to miR‐191‐5p. In A549 and H1650 cells, *SATB1* could upregulate the expression of β‐catenin, thus activating the Wnt/β‐catenin signaling pathway. Meanwhile, miR‐191‐5p could reduce the β‐catenin expression and the upregulation of *SATB1* could rescue this effect. Functional experiments indicated that upregulating *SATB1* could partially improve the inhibition of miR‐191‐5p on cell migration and proliferation. Combining the above results, we supposed that miR‐191‐5p might repress the *SATB1* expression and then partly inhibited the activation of Wnt/β‐catenin signaling pathway, thus leading to the impairment of cell proliferation and migration.

## 5 CONCLUSION

To sum up, it was found in this study that miR‐191‐5p could inhibit proliferation and migration of NSCLC cells, and its mechanism was probably to downregulate the *SATB1* expression, thus reducing the expression of β‐catenin, its downstream gene (Figure 7). This study might provide a new biomarker for detecting the disease and predicting its prognosis in the early stage as well as a therapeutic target in lung adenocarcinoma.

**Figure 7:** Graphical abstract of how miR‐191‐5p inhibits lung cancer. A schematic model of miR‐191‐5p/*SATB1*/β‐catenin pathway in lung cancer. miR‐191‐5p reduces the expression of *SATB1* and the level of β‐catenin

## CONFICT OF INTEREST

None.

## AUTHORS CONTRIBUTION

Fang Liu designed the research. Lai‐yong Zhou and Fu‐wei Zhang performed the experiments. Fang Liu and Jian Tong wrote the draft manuscript. All authors contributed to the writing and reviewing of the manuscript, and approved the final manuscript for submission.
